# Role of Intelligent Management Systems in Surgical Punctuality and Quality of Care

**DOI:** 10.1155/2022/4921644

**Published:** 2022-10-11

**Authors:** Gendi Li, Shenhui Huang

**Affiliations:** Operating Room of Huashan Hospital, Affiliated to Shanghai Fudan University Surgery, 200040 Shanghai, China

## Abstract

**Objective:**

The main objective is to illustrate the role of intelligent management systems in surgical punctuality and quality of care.

**Methods:**

72 registered nurses were selected from our operating room, and 180 patients who needed surgery were randomly divided into the control group and the observation group for satisfaction survey and satisfaction analysis.

**Results:**

The correct rate of surgical clothing distribution and the qualified rate of clothing recovery were improved, and the punctuality rate of the operation was enhanced than before the implementation of the intelligent management system. The accurate positioning of surgical items and the accurate statistics of equipment use time were enhanced than before implementation. The error rate of surgical item preparation after implementation was lessened than before implementation. Both nursing satisfaction and patient satisfaction after implementation were increased than before implementation.

**Conclusion:**

The intelligent management system improves the punctuality of surgery and the quality of care in the operating room.

## 1. Introduction

Operation room is usually involved in multiple departments which offer important treatment and rescue for patients. The patients admitted to the operation room are generally with serious diseases and complex situations, which require the high-quality nurses. Nurses play an essential role in the operating room work, and the health and safety of patients are closely related to the effectiveness of nursing in the operating room. Traditional operating room management mostly adopted manual recording which not only increases the work burden but also prone to mistakes. In addition, the risk of adverse events easily occurred due to the complexity of operating room nursing work. Strengthening nursing quality in the management of the operating room and standardizing the behavior and operation of nursing staff contribute to reducing the incidence of adverse events and improving the satisfaction rate of patients.

With the development of medical technology and the improvement of surgical quality requirements, the hospital management staff turning attaches importance to the master of operating room nursing technology to focus on the exploration of scientific management modes [1, 2]. Recently, the establishment of intelligent information in medical and health institutions throughout the country provides great convenience for medical staff. Moreover, the work efficiency of medical staff can be effectively improved based on the internet of intelligence and security [3]. As a new management mode, an intelligent management system has been employed to operating room work [4].

Intelligent operating room refers to the application of modern information technology in the operating room, and the use of high-tech software and hardware facilities can achieve modern operation process management [5]. The entry and exit of operating room medical staff can be obviously controlled by utilizing an information management system, which greatly reduces the wear of operating clothes and the operating cost of the hospital [6]. Moreover, the integration of all data in the operating room can significantly control the arrival time of medical staff in the operating room and improve the on-time opening rate [7]. Through the management of medical practices and transportation of medical supplies, the patient's intraoperative and postoperative conditions can be followed up in time, which is convenient for medical staff to adjust the treatment plan according to the different states of patients [8]. Comprehensive operating room multisystem information can achieve information integration, effectively manage the flow of people, logistics, and highly improve the operation efficiency and perioperative quality control management.

In the present study, the improvement effect of an intelligent process management system on work quality in the digital process of the operating room was explored and analyzed the changes in related work quality of medical staff and patients' job satisfaction before and after implementation.

## 2. Methods

### 2.1. Participants

The study was approved by the ethics committee of Huashan Hospital, which is affiliated with Fudan University in Shanghai. From June 2019 to September 2021, 72 registered nurses aged 22 to 55 years old with an average age of (35.69 ± 8.456) were selected from the operating room of our hospital. 17122 surgeries were collected and adopted the traditional management mode and the intelligent management system in the operating room, respectively. 180 surgical patients ranging from 20 to 70 years old with average ages of (47.68 ± 12.76) years old and (44.97 ± 11.48) years old were randomly divided into prior implementation group (control group) and after implementation group (observation group) to investigate for satisfaction. The control group included 53 males and 37 females, and the observation group included 57 males and 33 females. There was no statistical divergence in baseline data between the two groups.

### 2.2. Inclusion and Exclusion Criteria

Inclusion criteria were as follows: I) all nurses have professional qualification certificate; II) the nursing age was more than 1 year and had working experience in a general hospital; III) the nurses are all women; IV) the patients requiring surgery; V) all participants signed informed consent.

Exclusion criteria were as follows: I) further education nurses; II) the nursing age was lower than 1 year; III) nurses without working experience in general hospital; IV) patients who do not require surgery; V) patients who do not sign informed consent.

### 2.3. Methods of Management Modes

The control group intervened with traditional management. The traditional management mode mainly includes manual registration of the identity of surgical staff, entering and leaving the operating room, receiving surgical clothing, and other medical behaviors. Drugs, equipment, and dressings in the operating room are kept in fixed locations by special personnel and checked regularly. Sterilization items in the operating room were marked with sterilization dates. The number of surgical instruments was counted and recorded by operators, and the operating room nursing staff before and after the operation was to ensure the normal operation.

The observation group adopted the intelligent management system. (I) Surgical clothing management automation recorded operators' information to realize intelligent collection and recycling of clothes and shoes in the operating room. The management system tracked the washing and disinfection and used the status and inventory of surgical clothing and shoes in the operating room to remind logistics personnel to add or clean surgical clothing and shoes in time. At the same time, for efficient management level, the whole process of closed-loop management is required for surgical clothing and shoes. (II) Operation staff access control: intelligent identification of operating room medical staff strictly control the operating room irrelevant medical staff entry to effectively control the risk of infection in the operating room. (III) Operation staff behavior management: the combination of an intelligent management system and enterprise scheduling system accurately records the time point of medical staff entering and leaving the operating room to assure the on-time rate of operation. (IV) Operating room system management: according to the operating room management requirements, the historical data of the system reasonably are stored and maintained regularly to ensure the normal operation of all equipment. V) Operating room audit management: safety checked surgical instruments, medicines, blood transfusions, and consumables to form multidimensional knowledge database for data sharing.

### 2.4. Observation Indexes

- The qualified recovery rate of surgical clothing was observed before and after the implementation of the intelligent management system. The quality rate of clothing recovery = cases of qualified cases of clothing returning after surgery/cases of medical staff × 100%.
- Observed the on-time operation opening rate before and after the implementation of the intelligent system, with the operation starting at 8:30 as the standard.
- Discrepancy before and after the implementation of the operating room nursing quality: five assessment team members with more than 10 years of nursing experience were selected, and the hospital operating room nursing quality questionnaires were used to evaluate the operating room nursing quality, including aseptic operation, surgical instruments for qualified, sterile items based nursing management, nursing documents, and operation 5 projects. The percentage system was adopted for each item, and the higher the score, the higher the quality of nursing in the operating room.
- Contrasted the satisfaction of medical staff before and after implementation. The satisfaction of medical staff was evaluated by the self-made satisfaction questionnaire of our hospital, which mainly included three aspects: changing clothes flow schedule, operating room environment, and statistical reports. The total score of each aspect was 0 to 100, and the higher the score is, the higher the satisfaction will be.
- The patient satisfaction questionnaire made by the hospital was adopted. The total score was 100 points, very satisfied: 90 points, satisfied: 75–90 points, general: 60–75 points, and unsatisfied:<60 points.

### 2.5. Statistical Analysis

SPSS 22.0 software (SPSS Inc., Chicago, USA) was utilized for statistical analysis of the obtained data. The measurement data were displayed as (*X* ± *S*), and *t*-test was utilized for statistical analysis between the two groups. Counting data were displayed as rate (%), and divergence was performed by X^2^ test (Chi-square test). *P* < 0.05 was considered as a statistically notable divergence.

## 3. Results

### 3.1. Divergence between Correct Rate of Distributing Surgical Clothing and Qualified Rate of Clothing Recovery before and after Implementation

The correct rate of distributing surgical clothing and the qualified rate of clothing recovery were both higher than before the implemented intelligent management system, with statistical significance (*P* < 0.05), as shown in Table 1.

### 3.2. A Class III Adverse Event Is One That Does Not Result in Any Impairment of the Patient's Body or Function despite the Occurrence of False Facts

The on-time rate of operation starting after the implementation of the intelligent management system was higher than before implementation, and the divergences were statistically notable (*P* < 0.05). The detection of potential safety hazards after the implementation of the intelligent management system was higher than before implementation, and incidences of Class III adverse events were lower after implementation compared to before implementation, but the divergence was not statistically notable (*P* > 0.05) as shown in Table 2.

### 3.3. Divergence of Surgical Items and Equipment of Medical Staff in Operating Room

The accurate positioning of surgical items and the accurate statistics of equipment use time after the implementation of intelligent management system were higher than before implementation, and the divergences were statistically notable (*P* < 0.05). The prepared surgical items incorrectly were lower after implementation compared to before implementation (*P* < 0.05), while the sterile items expire was lower after implementation compared to before implementation but the divergence was not statistically notable (*P* > 0.05) as shown in Table 3.

### 3.4. Divergence of Nursing Quality before and after Implementation

The qualified preparation of equipment, qualified preparation of aseptic materials qualified, emergency supplies intact, and qualified nursing technique operation were higher than before implementation, and the divergences were statistically notable (*P* < 0.05) as shown in Table 4.

### 3.5. Discrepancy of Performance Appraisal Score of Operating Room Hospital

The work motivations of nurses were promoted after implementation compared to before implementation (*P* < 0.05). The job responsibility and the service attitudes were higher than before implementation; however, the divergences were without statistically notable (*P* > 0.05) as shown in Table 5.

### 3.6. Discrepancy of Satisfaction of Medical Staff before and after Implementation

The very satisfied number of nurses was more than before implementation, whereas the result did not reach statistical significance, and the divergences were statistically notable (*P* > 0.05). In addition, the satisfied number of nurses was more than before implementation, and the unsatisfied number of nurses was less than before implementation as shown in Table 6.

### 3.7. Discrepancy of Data between Control Group and Observation Group

180 surgical patients were randomly divided into control group and observation group. The control group included 53 males and 37 females, and the observation group included 57 males and 33 females. There was no statistical divergence in baseline data between the two groups as shown in Table 7.

### 3.8. Comparison of Satisfaction of Patients before and after Implementation

The very satisfied number of patients was more than before implementation, while the result did not reach statistical significance, and the divergences were statistically notable (*P* > 0.05). In addition, the satisfied number of nurses was more than before implementation, and the unsatisfied number of nurses was less more than before implementation as shown in Table 8.

## 4. Discussion

In recent years, due to the continuous improvement of people's living standards and the continuous development of medical technology, patients have higher requirements for the quality of surgery, especially for the surgical staff and surgical environment [9]. It is widely known that the more personnel entering the operating room, the greater the impact on the operating room environment. Therefore, the entry and exit of personnel in the operating room must be strictly controlled. The traditional setting of full-time personnel to check and register the medical staff participates in the operation and issues the key to the locker of changing clothes and shoes. With the gradual development of the intelligent operating room system, the introduction of information technology into operating room management has become the trend of operating room construction [10–13]. The intelligent surgical management system not only effectively controls the entry and exit of operating room personnel but also realizes the closed-loop tracking of surgical clothing [14]. The intelligent management system is of great help to the hospital to improve the regional management of operating room and standardize the behavior of medical staff [15].

The automatic and intelligent management of the distribution and recovery of operating clothes and shoes plays an important role in the management of the operating room [16]. Traditional operating room personnel receives surgical clothes and shoes through the manual record, while the surgical intelligent clothes sending machine is customized and developed based on the actual needs of the hospital. The dispensing machine is automatically associated with the operation schedule record of the hospital information system to realize the automatic dispensing of surgical clothes according to the size and effectively avoid the wrong dispensing of surgical clothes size [17]. The intelligent management system accelerated the turnover of surgical clothing via optimizing the changing process and simplified the counting process through the closed-loop tracking of washing, disinfection, receiving, and inventory of surgical clothing, which was more conducive to hospital logistics management [18]. What is more, the application of smart locker management also cultivated the habit of utilizing the wardrobe according to regulations and returning clothes in time, and the dressing recovery rate of medical staff was memorably boosted. The application of an intelligent management system not only lessened the workload of cleaning staff but also enhanced the satisfaction of medical staff to the changing process and operating room environment, bringing a better sense of experience to medical staff.

The on-time opening rate of operation is one of the indexes to evaluate the medical staff's behavior standard [19]. Before the application of the intelligent management system in the operating room, the operation is likely to be delayed due to the weak time concept of the operating room medical staff. In addition, there are often many and miscellaneous departments involved in the operation, and the operating room itinerant nurses often need to contact anesthesiologists and surgeons, which not only increases the working burden of the itinerant nurses but also increases the hidden danger of operation safety [20]. After the application of the intelligent management system, the intelligent management system plays a good reminder role for the operating room medical staff through the planning of the operating room time and the operation information push function and effectively improves the on-time operation opening rate. Meanwhile, it improves the management level and service level of the hospital operating room and further effectively improves the medical behavior of medical staff and the quality of work [21]. The operation desk information can be sent to the nurse station in the ward, which is beneficial for nurses to prepare related work in advance. The operation desk information can also be pushed by the operation desk information, which ensures that the operation doctors can get the operation desk information in time, so as to arrange the time and work reasonably and avoid the operation delay due to other work.

There are many kinds of equipment and sterile items in the operating room. In order to improve the precision of equipment management and timely statistics on the use, recovery, and storage of sterile items, the intelligent management system can scan these equipment and sterile items to realize information sharing [22]. This study shows that the intelligent management system has the function of recording and identifying, which can effectively manage sterile items and surgical equipment, accurately count the use time of equipment and sterile dressing cycle, and effectively reduce the expiration and failure rate of sterile items. At the same time, the intelligent management system has a verification function, which greatly reduces the incidence of medical errors, ensures the smooth development of surgery, and directly ensures the safety of surgery.

Intelligent management system to adhere to the quality improvement as the basic concept can improve the medical staff's work initiative and stimulate the sense of responsibility. This study shows that after the application of intelligent management system, the performance evaluation score is significantly improved, and the distribution of performance evaluation can be reasonably completed in a short time, which is conducive to improving the satisfaction of medical staff. In addition, an intelligent operating room can fully integrate patient information, ensure accurate operation, and reduce adverse events caused by improper operation of nursing staff, so as to ensure service quality and improve patient satisfaction.

## 5. Conclusion

Taken together, the efficiency of medical staff has been improved by intelligent management systems, which have changed the original manual management model. The intelligent management system can effectively improve the on-time operation opening rate, optimize the dressing process, improve the quality of nursing in the operating room, and reduce the occurrence of adverse events in the operating room, which is conducive to enhancing the satisfaction of medical staff and patients.

## Figures and Tables

**Table 1:** Divergence between the correct rate of distributing surgical clothing and qualified rate of clothing recovery before and after implementation (*n*, %).

Groups	Distribute surgical clothing correctly	Qualified rate of clothing recovery
Before implementation (*n* = 72)	66	58

After implementation (*n* = 72)	72	69
X^2^	6.261	8.07
P	0.028	0.004

**Table 2:** A Class III adverse event is one that does not result in any impairment of the patient's body or function despite the occurrence of false facts (*n*, %).

Groups	The on-time opening rate of operation	Occurrence of potential safety hazards	Class III adverse events
Before implementation (*n* = 8561)	7734	7	5

After implementation (*n* = 8561)	8063	15	2
X^2^	88.543	2.913	1.286
P	0.000	0.088	0.453

**Table 3:** Divergence of surgical items and equipment of medical staff in operating room (n, %).

Groups	Accurate positioning of surgical items	Sterile items expire	Prepare surgical items incorrectly	Accurate statistics ofequipment use time
Before implementation (*n* = 8561)	7138	9	13	7389

After implementation (*n* = 8561)	8096	4	3	8350
X^2^	546.348	1.925	6.256	726.444
P	0.000	0.267	0.021	0.000

**Table 4:** Divergence of nursing quality before and after implementation (n, %).

Groups	Equipment preparationqualified	Sterile articlesqualified	Emergencysupplies intact	Qualified nursing techniqueoperation
Before implementation (*n* = 8561)	8079	8417	8348	8481
After implementation (*n* = 8561)	8365	8520	8496	8533
X^2^	125.617	57.972	80.092	25.196
P	0.000	0.000	0.000	0.000

**Table 5:** Discrepancy of performance appraisal score of operating room hospital (n, %).

Groups	Work motivation	Job responsibility	Service attitudes
Before implementation (*n* = 72)	60	63	65
After implementation (*n* = 72)	69	70	68
X^2^	6.028	4.823	0.886
P	0.026	0.055	0.532

**Table 6:** Discrepancy of satisfaction of medical staff before and after implementation (n, %).

Groups	Very satisfied	Satisfied	General	Unsatisfied
Before implementation (*n* = 72)	9	20	30	13
After implementation (*n* = 72)	13	37	20	2
X^2^	0.352	4.947	3.064	9.005
P	0.647	0.03	1.115	0.003

**Table 7:** Discrepancy of data between control group and observation group (‾*X* ± *S*).

Groups	Age	Gender(male:female)
Before implementation (*n* = 90)	(47.68 ± 12.76)	53:37
After implementation (*n* = 90)	(44.97 ± 11.48)	57:33
P	0.136	0.541
X^2^	—	0.374

**Table 8:** Comparison of satisfaction of patients before and after implementation (n, %).

Groups	Very satisfied	Satisfied	General	Unsatisfied
Before implementation (*n* = 90)	21	29	26	14
After implementation (*n* = 90)	27	43	16	4
X^2^	1.023	4.537	3.106	6.173
P	0.4	0.048	0.112	0.023

## Data Availability

The datasets used and analyzed during the current study are available from the corresponding author upon reasonable request.
